# ERK1/2 Pathway Is Involved in the Enhancement of Fatty Acids from *Phaeodactylum tricornutum* Extract (PTE) on Hair Follicle Cell Proliferation

**DOI:** 10.1155/2020/2916104

**Published:** 2020-10-30

**Authors:** Lei Xiao, Xia Zhang, Zhiyi Chen, Yuting Li, Bing Li, Lin Li

**Affiliations:** ^1^School of Food Science and Engineering, Guangdong Province Key Laboratory for Green Processing of Natural Products and Product Safety, South China University of Technology, Guangzhou 510640, China; ^2^Infinitus (China) Co., China; ^3^Sericultural & Agri-Food Research Institute, Guangdong Academy of Agricultural Sciences, Key Laboratory of Functional Foods, Ministry of Agriculture and Rural Affairs, Guangdong Key Laboratory of Agricultural Products Processing, Guangzhou 510610, China; ^4^School of Chemical Engineering and Energy Technology, Dongguan University of Technology, College Road 1, Dongguan 523808, China

## Abstract

Extractions from *Phaeodactylum tricornutum* have been widely studied and evaluated to various biological effects. The aim of this study was to investigate the promotional effect of *P. tricornutum* extract (PTE) on the ERK1/2 signaling pathway involved in hair follicle cell proliferation. In order to illuminate the enhancement of PTE on hair growth by promoting proliferation of hair follicle cells, the activities of human hair follicle outer root sheath cell (HFORSC), human hair follicle germinal matrix cells (HFGMC), and hair epithelial melanocytes (HEM) were observed under PET treatment. Levels of keratins, PKC*ζ*, ERK1/2, and p38 MAPK in hair follicle cells were determined by Western blotting to illustrate the mechanisms of PTE effects on hair growth. Analyzed by GC-MS, the main polyunsaturated fatty acids which were 9.43% of total fatty acids in PTE were linolenic acid, linoleic acid, eicosapentaenoic acid, and docosahexaenoic acid. Melanin content and tyrosinase activity in HEM were measured. The results showed that PTE exhibited remarkable enhancement on cell proliferation. Melanin production was inhibited by PTE treatment, while keratin-14, keratin-15, and keratin-17 levels on hair follicle cells were elevated at different concentrations. The promotions of ERK1/2 and p38 MAPK levels indicated that the ERK1/2 signaling pathway is involved in the proliferation of hair follicle cells. These results are the evidence that PTE potentially deserves further study as a new natural candidate for hair care applications.

## 1. Introduction

*Phaeodactylum tricornutum* (*P. tricornutum*), an interesting natural material, is a common type of marine diatoms with three different morphotypes, of which the genomes have been fully sequenced [1]. *P. tricornutum* constituents with multiple components such as proteins, carotenoids like fucoxanthin, polyphenols like (epi-)catechin, vitamins, minerals, and several kinds of lipophilic materials of polyunsaturated fatty acids (PUFAs), such as eicosapentaenoic acid (EPA) and docosahexaenoic acid (DHA), which might mediate physiological values [2–6].

The antioxidant capacity, cytotoxicity, immunomodulatory activity, and antimicrobial ability, as well as antiobesity and antidiabetic properties of the extractions from *P. tricornutum* (PTE) have been widely studied and evaluated. PTE showed abilities to stimulate proteasome activity on human keratinocytes under UVA and UVB radiations, as evidence indicated that carbonyl content of total protein and oxidized protein level was reduced in PTE-treated cells both before and after UV irradiation to further preserve proteasome function in lowering the irradiation-induced protein oxidative damage [7]. PET also showed the capability to have protective effects on protein oxidation level in human stratum corneum post UVA and UVB exposures [8]. There are publications and patents that archived PTE antioxidation and proteasome peptidase activities from the detrimental effects of UV exposure [9]. Beneficial effects such as anti-inflammation were evaluated [10, 11]. New compounds, such as carotenoid, from PTE exhibited health benefit effects of inflammatory reduction, alleviation of oxidative stress, and interference with cancer cells [12]. PTE, rich with fucoxanthin, comprises several lipophilic constituents and showed antiobesity and antidiabetic properties that have been reported in cell and in vivo studies [13–15]. The antiobesity effects of *ω*-3 long-chain PUFAs comprise decreased lipogenesis and the enhancement of fatty acid oxidation in liver and adipose tissues, as well as the influence of intestinal lipid absorption and lipid metabolism [16, 17]. As the result, the interesting properties of PTE were described above and further studies on PTE-related biological effects may lead to important clinical as well as economic significances.

Hair, as the skin appendage growing on the surface of the scalp with its appearance and protective functions, has been considered to play important roles in human daily maintenance. The human hair follicle (HF) is highly dynamic that repeatedly and perpetually undergoes tightly programmed cyclical transformations through periods of active hair growth (anagen), apoptosis-driven involution (catagen), hair shedding (exogen), and relative resting (telogen) [18, 19]. During HF growth and hair production, the activity of factors promoting the proliferation, differentiation, and survival predominates, whereas HF regression is characterized by the activation of a variety of signaling pathways that induce apoptosis in HF cells [20]. Continuation and transition of each phase of hair growth result from elaborate interactions between mesenchymal dermal papilla, located at the base of the hair follicle, and adjacent follicular epithelium.

Hair problems, such as hair loss and grey hair, may result from hair cell imbalances of metabolisms or outer injuries of physical and chemical interferences. The regeneration and self-healing of HF are vital in maintaining normal hair growth. Among the follicular epithelium are HF outer root sheath cells (HFORSC) that form the HF and are the repairmen of epidermis cells [18]. HF germinal matrix cell (HFGMC), located at the base of the bulb and the main source for hair growth, goes through cornification to form a layer of keratin to suppress hair loss. And HF inner root sheath cells (HFIRSC) keep the hair steady in HF. In particular, mesenchyme-derived dermal papilla cells (DPC) have potential to induce hair follicle formation [21]. A number of signals from DPC may directly influence HFORSC in the bulge area to regulate hair growth cycle [22]. Besides, keratins including keratin-14, keratin-15, keratin-17, and keratin-19 related to HFORSC have properties in the formation of HF [23]. Hair pigmentation is coupled to the HF growth cycle that occurs only during anagen and stops very early in the anagen-catagen transition [24]. Tyrosinase is detected in hair bulb melanocytes, pointing to a melanin-producing subpopulation of the follicular melanocytes, while the mechanism of the pigment incorporating into the hair shaft or being removed from the hair bulb during early catagen is not clear [25, 26]. Epidermal hairs are usually nursed by hair care routines. However, some of the routines could contribute to some degrees of hair problems.

It would be meaningful to find better materials or routines with less damage on hair growth. Some natural extracts have been believed to regulate hair cell growth with less damage on HF cells. In order to obtain better insight into the possible benefits of PTE influences on human hair growth, we focused on its biological effect on HF cell growth, level of key protein including keratin, and HF cell-related melanin production. This work will be helpful in broadening ideas for future investigations of PTE on hair care applications.

## 2. Results

### 2.1. Influences of PTE on Hair Follicle Cell Viability and Growth

The influences of PTE on HFORSC, HFGMC, and HEM proliferations were evaluated with MTT assays. Cells were treated with serial dilutions of PTE at the range from 0.03 *μ*g/mL to 16 *μ*g/mL in correspondent culture media for 24 hours at 37°C in a CO_2_ incubator. The results showed significant reduction effect on both HFORSC and HFGMC proliferations at higher concentrations between 4 *μ*g/mL and 16 *μ*g/mL, while there was statistical significance of cell growth-promoting effects on both HFORSC and HFGMC proliferations at lower concentrations ranged from 1 *μ*g/mL to 2 *μ*g/mL in comparison with their control (Figures 1(a) and 1(b)). The proliferation of HEM was not affected by PTE treatment at concentrations ranged from 1 *μ*g/mL to 8 *μ*g/mL but was significantly induced at concentrations ranged from 0.125 *μ*g/mL to 0.5 *μ*g/mL (Figure 1(c)). This result may indicate that PTE exhibited some kind of promoting effects on proliferation of hair follicle cells.

Cell colony formation is a primmorph counting of the proliferation from single cell in vitro. The adaption ability of a colony is stronger than the single cell under signals or stimulations. A colony forming experiment is a kind of test to challenge individual cells under low cell density, which shows higher sensibility in analyzing the cell viability. Statistical data of stained colonies are presented in Figure 1(d). It showed a significant rise of the HFGMC colony formation at 0.125 *μ*g/mL of PTE, while a significant increase of the HFORSC colony formation at 0.0625 *μ*g/mL. PTE at other concentrations could also raise the colony numbers but showed no statistical significances. The results indicated that PTE could enhance the colony multiplications on HFORSC and HFGMC, especially at concentration ranges from 0.0625 *μ*g/mL to 0.125 *μ*g/mL.

In order to evaluate long-term influences of PTE effects on hair follicle cells, the growth profiles of HFORSC and HFGMC were evaluated under PTE treatment with the concentration of 0.0625 *μ*g/mL obtained from cell colony formation assay. The results showed that there was no significant difference in cell growth levels between the PTE-treated group and the control group on both cells (Figures 1(e) and 1(f)), which indicates that PTE has no long-term effect on the growth of hair follicle cells at low concentrations.

### 2.2. Influences of PTE on Keratin Level

Keratins, expressed in HFORSC and dermal papilla, are the main components of the cortex and medulla, which have great influences on hair structural strength and thickness, where keratin-15 and keratin-19 are epidermal stem signs that reflect the cell abilities of differentiation and proliferation. Influences of PTE on HFORSC keratin-14, keratin-15, keratin-17, and keratin-19 were examined (Figure 2). The results indicated that expression levels of keratin-14, keratin-15, and keratin-17 in HFORSC were enhanced with PTE at various concentrations. There were significant increases of 77%, 49%, and 131% in keratin-14, keratin-15, and keratin-17, respectively, with PTE at 0.25 *μ*g/mL.

### 2.3. Influences of PTE on Melanin Production and Tyrosinase Activity of HEM

In this experiment, 8-methoxypsoralen (8-MOP) was chosen as a positive control since it is photosensitive with melanin-promoting and tyrosinase-activating abilities. PTE treatment groups had no melanin inductions in the treatment concentrations but exhibited melanin reduction significantly at concentrations of 0.25 *μ*g/mL and 0.50 *μ*g/mL, as well as the 8-MOP treatment had melanin-promoting abilities on HEM (Figure 3(a)). On the other hand, tyrosinase activities were significantly induced with the PTE treatment at concentrations of 0.125 *μ*g/mL, of which the tyrosinase activity was higher than the 8-MOP treatment group (Figure 3(b)), although the melanin level showed no significant differences with PTE treatment at the same concentration.

### 2.4. Influences of PTE on ERK1/2, p38, and PKC*ζ* Expression in HEM

It has been reported that the activation of extracellular signal-regulated kinase (ERK) reduces melanin synthesis, as well as the inhibition of p38 MAPK (mitogen-activated protein kinase) blocks melanogenesis [27]. Protein kinase C zeta (PKC*ζ*) activation plays a predominant role in the formation of melanocyte dendricity [28]. Influences of PTE on HEM protein expressions of ERK1/2, p38 MAPK, and PKC*ζ* are presented in Figure 4. The expressions of ERK1/2 were induced by 56% with PTE treatment at a concentration of 0.5 *μ*g/mL, while the expression level of p38 MAPK exhibited an insignificant increase at about 17%. PTE treatment showed no significant influence on PKC*ζ* expression levels in HEM at all tested concentrations.

## 3. Discussion

### 3.1. Enhancement of PTE on Hair Follicle Cell Growth

Hair follicle is composed of the epithelium and leather parts. The epithelial part includes the inner root sheath and outer root sheath. The leather part includes the dermal papillae and dermal sheath, of which the morphology of hair follicle generation is induced by interactions of the epidermis and dermis. The cyclicality stages of hair growth includes anagen, catagen, telogen, and exogen, and the cyclic growth cycles repeat the hair follicle's whole life [29]. The outer root sheath cells which are composed by a large number of undifferentiated cutin with long proliferation cycle and stem cell properties are involved in the formation of the hair follicle and repairmen of epidermis cells [27]. The inner root sheath cells are the one layer of cells that cling to hair, which play an important role in keeping the hair steady in the hair follicle. HFGMC, located at the base of the hair bulb around the nipples, is the main support for hair growth and hair melanin transfer. In the active stages of hair growth, quick cell growth and differentiation contribute to hair growth. HFGMC goes through cornification to form a layer of keratin to suppress hair loss. During the cyclicality, all of the above mentioned cells interact with each other to support the growth of hair. In our current studies, the HFORSC and HFGMC were chosen to evaluate the PTE abilities to influence on hair follicle regeneration and hair growth.

HFORSC is connected with epidermal basal layer cells anatomically that is widely accepted to have the characteristics of stem cells, while HFGMC is considered as the main resource of hair growth [30]. Cell viability study results indicated that PTE treatments could effectively increase the proliferation abilities on HFORSC and HFGMC at concentrations from 0.0625 *μ*g/mL to 0.125 *μ*g/mL. Therefore, PTE effects on HFORSC and HFGMC proliferation inductions could possibly relate to influence on hair follicle proliferation and hair growth.

### 3.2. Influences of PTE on Keratin Level in Hair Follicle Cell

Keratins of the cortex are essential factors to support the tenacity and elasticity of hair. Thus, the general hair quality is believed to have some correlations to the keratin levels of HFORSC and HFIRSC. Keratin-14, a type I keratin in normal epidermis which is mainly expressed in the basal layer cell with fission and proliferation abilities, is of great importance in maintaining the proliferation and differentiation of skin basal layer cells and the integrity of cell morphology [31, 32]. Keratin-15, as a sign of hair follicle stem cells, is specifically expressed in HFORSC [33]. Keratin-19 is generally considered as one of the symbols of epidermal stem cells. The self-renewal, proliferation, and differentiation abilities of cells could be implied by its expression level. Keratin-15 and keratin-19 are remarkably expressed in the gathering area of epidermal stem cells and hair follicle outer root sheath uplift area (bulge) [34]. Previous research showed that keratin-15 and keratin-19 have no expression in vitro generation of cultured HFORSC, which implies loose of differentiation ability [35]. PTE enhanced various degrees of protein expressions of keratin-14, keratin-15, and keratin-17 on HFORSC in this study (Figure 2) which could be a possible indication that PTE is involved in regulating hair tenacity and elasticity. Further, the increased protein expression levels of keratin-14, keratin-15, and keratin-17 on HFORSC under the treatments of PTE might indicate regulatory effects at molecular levels to improve the renewals of hair follicle and hair growth based on the mechanisms of proliferation and differentiation.

So far, there were studies that indicated a total of 54 kinds of keratins in human beings, 37 of which exist in the epithelial cell and 17 kinds in the hair. Furthermore, 9 keratins are specifically expressed in hair follicle epithelial cells. As a main component of the cytoskeleton, hair follicle keratins are of great importance in keeping the mechanical stability and integrity of the epithelial cell as well as the structure of hair follicles [33]. There are 5 kinds of hair follicle keratins related to hereditary hair disorders [36]. Among them, there were lots of attention on keratin-17, a kind of keratin which supports the structure of cells and could promote the hair follicle growth by reducing the TNF-*α*-induced apoptosis [37]. Mice lacking keratin-17 had severe moulting, brittle hair, apoptosis of hair follicle stromal cells, and hair follicle histology change [38]. The expression of keratin-17 could be easily induced in stratified epithelial cells to regulate the growth of the cells and renovation of the skin [39]. In this study, a 131% expression level increase of keratin-17 on HFORSC by PTE indicated that PTE could act as an enhancer to influence hair follicle activities effectively and act as a protector to maintain hair normal structure.

### 3.3. Influences of PTE on Melanogenesis

The synthesis of melanin initiates in mature melanocytes in the hair follicle active growth phase, and then the melanin were transferred into the hair cortex. The cellular tyrosine is catalyzed by tyrosinase into the molecules of Dopa and then Dopaquinone. Thus, the activity of tyrosinase could be an indicator to predict melanin formation following melanosome transfer of melanin into horn cells by synapse regulated by signal PKC*ζ*. On the other hand, melanin level could be inhibited by activation of the ERK pathway [27]. The current study showed that the activity of tyrosinase, the expression level of ERK1/2, and the melanin levels in HEM cells were all influenced by PTE. A study showed that PTE concentrations at 0.125 *μ*g/mL to 0.5 *μ*g/mL could significantly increase the proliferation of HEM (Figure 1(c)), but the development of melanin is inhibited (Figure 3(a)). The promotions of melanophore and tyrosinase are supposed to bring increases of melanin level, but our current study showed melanin decrease and tyrosinase increase induced by PTE at 0.125 *μ*g/mL. Established cocultures of melanocytes and keratinocytes could provide a closer model to the body physiological state to understand the interactions between melanophore and keratinocyte [40]. Therefore, PTE speculations on melanin metabolisms could be further evaluated with the coculture method.

PKC*ζ* is a vital regulator of synapse formation of the 5 kinds of PKC subtypes expressed by melanophore, especially prostaglandin E2 [28]. The mitoses, cell polarity, and differentiation are all managed by PKC*ζ*. A study indicated that the activation of PKC*ζ* could also increase the development of synapses and transfer the amount of melanosome into adjoining cells [41]. Our current experiment showed less significance of the PTE effect on the PKC*ζ* level (Figure 4). This result might be a biological benefit with the maintenance of normal expression of PKC*ζ*, which is of great importance to normal metabolism without overexpression of PKC*ζ* that could trigger tumors [42].

ERK1/2, which is related to cell proliferation and apoptosis, is a main pathway of MAPK pathways. Research had proven that the activation of ERK and Akt could protect the Mel-Ab cells from the apoptosis induced by UVB [43]. Other studies found that the activation of ERK could inhibit the activity of melanin enzyme and generation of melanin [44, 45]. Kim et al. chose the human melanophore as a material and concluded that the activation of ERK and inhibition of p38 MAPK could both reduce the generation of melanin [27]. Our current study showed that PTE promoted 56% of the ERK1/2 level (Figure 4) which was was consistent with the reduction of the melanin level. The level of p38 MAPK was slightly increased but had no significant influence on the generation of melanin. Considering the PTE influences on promotions of the level of ERK1/2 and p38 MAPK, and the enhancement of HEM growth, we believed that melanogenesis could be regulated by PTE at proper concentrations.

## 4. Conclusions

The liposoluble extract from *Phaeodactylum tricornutum* exhibited activities on hair growth by promoting the growth of hair follicle cells and showed influence on the melanogenesis in melanophore. Thus, this extract could provide a new natural compound for hair care applications by regulating hair cell growth.

## 5. Methods

### 5.1. Materials

*P. tricornutum* was collected from a salted lake and isolated by the South Central University for Nationalities in China. The cultivation was conducted in a modified f/2 medium and lasted for 10 days. Then, the microalgal cells were harvested by centrifuge and freeze-dried for extraction. To prepare the PTE extract, disperse 20 g of frozen dry mass in 500 mL of 95% ethanol rendered alkaline to pH 13 by adding 30% aqueous sodium hydroxide solution. Reflux at 79°C for 30 min under a nitrogen atmosphere and cool to 18°C. Remove the insoluble materials by filtration. Add 150 mL distilled water and agitate to form an aqueous-alcoholic phase. Wash the aqueous-alcoholic phase with heptane by a liquid-liquid process and get the lower phase. Repeat two times and acidify the lower phase to a pH value of 2.5 by the addition of sulfuric acid. Wash with heptane three times. Remove heptane with a rotary evaporator to get 0.197 g of PTE extract with dark yellow oily appearance.

Dulbecco's modified Eagle's medium (DMEM) with high glucose, fetal bovine serum (FBS) and cell culture supplements of penicillin, streptomycin, and L-glutamine were purchased from Gibco® Life Technologies. Cell culture disposable sterile materials with the name brand of Corning® were purchased from Thermo Fisher. Mouse anti-cytokeratin 14 monoclone antibody (Ab49806), rabbit anti-cytokeratin 15 monoclone antibody (Ab139840), and rabbit anti-KRT71 polyclone antibody (Ab133817) were purchased from Abcam; mouse anti-cytokeratin 19 monoclone antibody (Sc-374192), mouse anti-cytokeratin 17 monoclone antibody (Sc-393091), and rabbit anti-PKC*ζ* polyclonal serum (Sc-216) were purchased from Santa Cruz Biotechnology; and rabbit anti-P44/42 MAPK (ERK1/2) monoclonal antibody (CST#4695), rabbit anti-tubulin monoclonal antibody (CST#2125), and rabbit anti-p38 MAPK (D13E1) monoclonal antibody (CST#8690) were purchased from Cell Signaling Technology. The PTE extract was prepared by the methods of Nizard et al. with some modification as indicated above [9]. 3-(4,5-Dimethyl-2-thiazolyl)-2,5-diphenyl-2-H-tetrazolium bromide (MTT), dimethyl sulfoxide (DMSO), Nonidet P-40, L-3,4-dihydroxyphenylalanine (L-Dopa), 8-methoxypsoralen (8-MOP), and other chemical reagents, if not specified, were purchased from Sigma-Aldrich Co.

### 5.2. Determination of Fatty Acid Composition of PTE

Derivatization of fatty acids in PTE was prepared by the transesterification method [46]. Then, the fatty acid methyl esters were analyzed by GC-MS. Decanoic acid methyl ester was used as the internal standard. Samples were analyzed by using Agilent Technology 7820A GC and 5977E MSD systems equipped with an autosampler. Chromatographic separations were carried out by using a TG-Wax MS column (Thermo Scientific™) with 30 m length, 0.25 mm internal diameter, and 0.25 *μ*m column phase thickness. Nitrogen was used as carrier gas, and 1 *μ*g volume of the sample was injected to the inlet heated to 280°C with a splitless injection mode. The oven temperature was programmed at 120°C initially and held for 3 min and raised up to 240°C at a speed of 5°C/min, until it reaches 240°C with an 8 min hold time. Conditions used for the mass spectrometer were a source temperature of 230°C, scan range 40-650 m/z, and operation in positive electron impact mode with ionization energy of 70 eV. Chromatographic and mass spectral data were analyzed by the instrument built in MSD ChemStation (Agilent Technologies, USA). Quantification of fatty acids was calculated by the internal standard with the relationship of relative response factors. The result showed that PTE contained a unique fatty acid profile (Table 1), especially some polyunsaturated fatty acids such as linolenic acid (C18:3n3), linoleic acid (C18:2n6c), eicosapentaenoic acid (EPA, C20:5), and docosahexaenoic acid (DHA, C22:6).

### 5.3. Cell Cultures

HFORSC, HFGMC, and HEM were bought from Beijing Yuhengfeng Biotech Co., Ltd. Before incubating, epidermal growth factor and mesenchymal stem cell growth factor are added to stabilize cell amplifications in the culture media. The cells were maintained and cultivated in DMEM containing 10% FBS, with 5% CO_2_ at 37°C. Cells from the third to sixth passages of subcultures were used for experiments.

### 5.4. MTT Assay for Cell Viability and Proliferation

Influence of PTE on cell proliferations was measured by the MTT method as previously described [47]. PTE extract was sterilized by filtration with 0.22 *μ*m microporous membrane and diluted with culture media containing 10% FBS to have an initial concentration of 16 *μ*g/mL. The media of cell cultures at 80% confluence in 96-well cell culture plates were replaced by the PTE serial dilutions, respectively, with 5 parallel wells at each concentration. MTT assays were conducted on the cells after 24-hour treatments with PTE dilutions. The results were expressed as a percentage of the untreated controls, and the values were represented as the mean ± SD.

### 5.5. Colony Formation Test and Cell Growth Curve

Inoculate HFORSC and HFGMC into a 6-well plate at concentrations of 2.00 × 10^2^ cells per well and 5.00 × 10^2^ cells per well, respectively. The cell culture media were replaced with PTE dilutions at 0.0625 *μ*g/mL, 0.125 *μ*g/mL, and 0.25 *μ*g/mL after the cell adhering onto the bottom of the plates with 3 parallel wells of each concentration. After 6-day incubation at 37°C with 5% CO_2_, cells were stained with 5% crystal violet for 4 hours, the excessive dye was washed away with PBS, and the cell colonies were counted under a light microscope.

2 mL of HFORSC and HFGMC cell culture suspension (about 2.25 × 10^4^ cells/mL) was inoculated into a 3.5 cm culture dish. The culture media was replaced with PTE at a concentration of 0.0625 *μ*g/mL after the cultured cell adhered onto the bottom of the culture dish. Cell numbers were counted every day for six days in order to establish the cell growth curves.

### 5.6. Western Blotting

HF cells were incubated in culture media with 10% FBS until the cell culture was at 30% in confluence in the culture dish. The culture media were replaced with the PTE dilutions at the concentrations of 0.125 *μ*g/mL, 0.25 *μ*g/mL, and 0.5 *μ*g/mL with proper controls and incubated at 37°C with 5% CO_2_ until the cell culture reached at 80% confluence. The level of keratin and other proteins in cells was assessed by Western blot. Proteins were extracted by cracking cells in a lysis buffer with protease inhibitors on ice. The protein concentration was adjusted to the same level by Bradford assay before being loaded in the SDS-PAGE. *α*-Tubulin was used as an internal control to normalize other protein expression levels in this experiment. The densities of the protein images from Western blots were quantified by the software ImageJ and normalized in comparison to the internal control protein of *α*-tubulin to determine the protein levels.

### 5.7. Measurements of Melanin Levels and Tyrosinase Activities

When the HEM cell cultures were at 20% in confluence, the culture media were replaced with media containing PTE at different concentrations and 8-MOP at 10 *μ*mol/L, respectively. The HEM were incubated until the cultured cells reached 90% in confluence at 37°C with 5% CO_2_. The cultured cells were trypsinized and washed twice with PBS at 6,000 g centrifugations. For the melanin level determination, the cell numbers were adjusted and pelleted at 1.00 × 10^6^ cells per sample for melanin level measurements with 0.5 mL NaOH (1N) resuspension following 30-minute incubations at 60°C in a water bath. The NaOH cell suspensions were measured with a chroma meter at 405 nm for melanin levels. For the tyrosinase activity measurement, the cell numbers were adjusted and pelleted at 2.00 × 10^5^ cells per sample. The extraction buffer containing 1% Nonidet P-40, 0.01% SDS, and proteinase inhibitors (3 *μ*g/mL aprotinin, 2 *μ*g/mL pepstatin, 1 *μ*g/nL leupeptin, 0.1 *μ*M PMSF, and 1 mM DTT) was added into each sample and treated by ultrasound at 4°C for 5 minutes following a 30-minute centrifugation at 12,800 g to obtain supernatants as the tyrosinase is extracted. The tyrosinase activity was measured with the absorbance at 492 nm after mixed 70 *μ*g tyrosinase extracts and 100 *μ*g L-Dopa at 37°C for 30 min.

### 5.8. Statistical Analysis

All values are presented as means ± standard deviations (SD) of triplicate samples. Differences between two groups were assessed using unpaired two-tailed Student's *t*-test. In all statistical comparisons, *P* < 0.05 was defined as significant. GraphPad Prism software was used for all calculations.

## Figures and Tables

**Figure 1:** Influences of PTE on cell viability and growth of HFORSC, HFGMC, and HEM. (a–c) Proliferation activities of HFORSC, HFGMC, and HEM determined by MTT assay; (d) colony formations of HFORSC and HFGMC; (e, f) long-term influences of PTE at 0.0625 *μ*g/mL on HFORSC and HFGMC growth. PTE: extractions from *Phaeodactylum tricornutum*; HFORSC: outer root sheath cells of human hair follicle; HFGMC: germinal matrix cell of human hair follicle; HEM: hair epithelial melanocytes. ^∗^*P* < 0.05 versus non-PTE-treated controls.

**Figure 2:** Influences of PTE on protein levels of keratin-14, keratin-15, keratin-17, and keratin-19 in HFORSC. (a) Western blot of keratin-14, keratin-15, keratin-17, and keratin-19 with PET treatment at concentrations of 0.0625, 0.125, and 0.25 *μ*g/mL; (b) normalized densities of keratin-14, keratin-15, keratin-17, and keratin-19 by ImageJ. PTE: extractions from *Phaeodactylum tricornutum*; HFORSC: outer root sheath cells of human hair follicle. ^∗^*P* < 0.05 versus non-PTE-treated controls.

**Figure 3:** Influence of PTE on melanin levels and tyrosinase activity of HEM. (a) Melanin levels; (b) tyrosinase activity. PTE: extractions from *Phaeodactylum tricornutum*; HEM: hair epithelial melanocytes; 8-MOP: 8-methoxypsoralen. ^∗^*P* < 0.05 versus non-PTE-treated controls.

**Figure 4:** Influences of PTE on protein levels of ERK1/2, p38 MAPK, and PKC*ζ* in HEM. (a) Western blot of ERK1/2, p38, and PKC*ζ* with PET treatment at concentrations of 0.125, 0.25, and 0.5 *μ*g/mL; (b) normalized densities of ERK1/2, p38, and PKC*ζ* by ImageJ. PTE: extractions from *Phaeodactylum tricornutum*; HEM: hair epithelial melanocytes. ^∗^*P* < 0.05 versus non-PTE-treated controls.

**Table 1:** Fatty acids profile of *Phaeodactylum tricornutum* extract determined by GC-MS.

	Fatty acids	Structure	Relative content (%)
1	C12:0		10.99
2	C14:0		7.874
3	C16:0		26.43
4	C16:1		34.45
5	C18:0		1.555
6	C18:1n9c		5.034
7	C18:2n6c		3.491
8	C18:3n3		0.507
9	C20:5		5.127
10	C22:1n9		0.695
11	C22:6		0.303
12	C24:0		2.72
13	C24:1		0.825

## Data Availability

All data included in this study are available upon request by contact with the corresponding author.

## References

[1] Bowler C., Allen A. E., Badger J. H. (2008). The Phaeodactylum genome reveals the evolutionary history of diatom genomes. *Nature*.

[2] Derwenskus F., Metz F., Gille A. (2019). Pressurized extraction of unsaturated fatty acids and carotenoids from wet Chlorella vulgaris and Phaeodactylum tricornutum biomass using subcritical liquids. *GCB Bioenergy*.

[3] Kim S. M., Jung Y. J., Kwon O. N. (2012). A potential commercial source of fucoxanthin extracted from the microalga Phaeodactylum tricornutum. *Applied Biochemistry and Biotechnology*.

[4] Sorensen M., Berge G. M., Reitan K. I., Ruyter B. (2016). Microalga Phaeodactylum tricornutum in feed for Atlantic salmon (Salmo salar) —effect on nutrient digestibility, growth and utilization of feed. *Aquaculture*.

[5] Foo S. C., Yusoff F. M., Ismail M. (2017). Antioxidant capacities of fucoxanthin-producing algae as influenced by their carotenoid and phenolic contents. *Journal of Biotechnology*.

[6] Rico M., Lopez A., Santana-Casiano J. M., Gonzalez A. G., Gonzalez-Davila M. (2013). Variability of the phenolic profile in the diatom Phaeodactylum tricornutum growing under copper and iron stress. *Limnology and Oceanography*.

[7] Bulteau A. L., Moreau M., Saunois A., Nizard C., Friguet B. (2006). Algae extract-mediated stimulation and protection of proteasome activity within human keratinocytes exposed to UVA and UVB irradiation. *Antioxidants & Redox Signaling*.

[8] DeGrey A. D. N. (2004). *Strategies for Engineered Negligible Senescence: Why Genuine Control of Aging May Be Foreseeable*.

[9] Nizard C., Friguet B., Moreau M., Bulteau A., Saunois A. Use of phaeodactylum algae extract as cosmetic agent promoting the proteasome activity of skin cells and cosmetic composition comprising same.

[10] Serini S., Bizzarro A., Piccioni E. (2012). EPA and DHA differentially affect in vitro inflammatory cytokine release by peripheral blood mononuclear cells from Alzheimer's patients. *Current Alzheimer Research*.

[11] Kim K. N., Heo S. J., Yoon W. J. (2010). Fucoxanthin inhibits the inflammatory response by suppressing the activation of NF-*κ*B and MAPKs in lipopolysaccharide-induced RAW 264.7 macrophages. *European Journal of Pharmacology*.

[12] Neumann U., Derwenskus F., Flister V. F., Schmid-Staiger U., Hirth T., Bischoff S. C. (2019). Fucoxanthin, A Carotenoid Derived from Phaeodactylum tricornutum Exerts Antiproliferative and Antioxidant Activities In Vitro. *Antioxidants*.

[13] Gille A., Stojnic B., Derwenskus F. (2019). A Lipophilic Fucoxanthin-Rich Phaeodactylum tricornutum Extract Ameliorates Effects of Diet-Induced Obesity in C57BL/6J Mice. *Nutrients*.

[14] Flachs P., Rossmeisl M., Kopecky J. (2014). The effect of n-3 fatty acids on glucose homeostasis and insulin sensitivity. *Physiological Research*.

[15] Maeda H. (2015). Nutraceutical effects of fucoxanthin for obesity and diabetes therapy: a review. *Journal of Oleo Science*.

[16] Woo M. N., Jeon S. M., Shin Y. C., Lee M. K., Kang M. A., Choi M. S. (2009). Anti-obese property of fucoxanthin is partly mediated by altering lipid-regulating enzymes and uncoupling proteins of visceral adipose tissue in mice. *Molecular Nutrition & Food Research*.

[17] Jang W. S., Choung S. Y. (2013). Antiobesity Effects of the Ethanol Extract of *Laminaria japonica* Areshoung in High-Fat-Diet-Induced Obese Rat. *Evidence-Based Complementary and Alternative Medicine*.

[18] Paus R., Cotsarelis G., Engl N. (1999). The Biology of Hair Follicles. *Journal of Medicine*.

[19] Cotsarelis G., Millar S. E. (2001). Towards a molecular understanding of hair loss and its treatment. *Trends in Molecular Medicine*.

[20] Soma T., Ogo M., Suzuki J., Takahashi T., Hibino T., Invest J. (1998). Analysis of Apoptotic Cell Death in Human Hair Follicles *In Vivo* and *In Vitro*. *Journal of Investigative Dermatology*.

[21] Jahoda C. A. B., Horne K. A., Oliver R. F. (1984). Induction of hair growth by implantation of cultured dermal papilla cells. *Nature*.

[22] Cotsarelis G., Sun T. T., Lavker R. M. (1990). Label-retaining cells reside in the bulge area of pilosebaceous unit: implications for follicular stem cells, hair cycle, and skin carcinogenesis. *Cell*.

[23] Langbein L., Yoshida H., Praetzel-Wunder S., Parry D. A., Schweizer J., Invest J. (2010). The Keratins of the Human Beard Hair Medulla: The Riddle in the Middle. *Journal of Investigative Dermatology*.

[24] Seiberg M. (2013). Age-induced hair greying - the multiple effects of oxidative stress. *International Journal of Cosmetic Science*.

[25] Commo S., Bernard B. A. (2000). Melanocyte subpopulation turnover during the human hair cycle: an immunohistochemical study. *Pigment Cell Research*.

[26] Tobin D. J. (2002). A possible role for Langerhans cells in the removal of melanin from early catagen hair follicles. *The British Journal of Dermatology*.

[27] Kim D. S., Park S. H., Kwon S. B., Na J. I., Huh C. H., Park K. C. (2007). Additive effects of heat and p38 MAPK inhibitor treatment on melanin synthesis. *Archives of Pharmacal Research*.

[28] Scott G., Fricke A., Fender A., McClelland L., Jacobs S. (2007). Prostaglandin E2 regulates melanocyte dendrite formation through activation of PKC*ζ*. *Experimental Cell Research*.

[29] Booth C., Potten C. S., Invest J. (2000). Keratinocyte Growth Factor Increases Hair Follicle Survival Following Cytotoxic Insult. *Journal of Investigative Dermatology*.

[30] Magerl M., Kauser S., Paus R., Tobin D. J. (2002). Simple and rapid method to isolate and culture follicular papillae from human scalp hair follicles. *Experimental Dermatology*.

[31] Yoshida K., Sato K., Tonogi M., Tanaka Y., Yamane G. Y., Katakura A. (2015). Expression of cytokeratin 14 and 19 in process of oral carcinogenesis. *The Bulletin of Tokyo Dental College*.

[32] Alam H., Sehgal L., Kundu S. T., Dalal S. N., Vaidya M. M. (2011). Novel function of keratins 5 and 14 in proliferation and differentiation of stratified epithelial cells. *Molecular Biology of the Cell*.

[33] Moll R., Divo M., Langbein L. (2008). The human keratins: biology and pathology. *Histochemistry and Cell Biology*.

[34] Lyle S., Christofidou-Solomidou M., Liu Y., Elder D. E., Albelda S., Cotsarelis G. (1998). The C8/144B monoclonal antibody recognizes cytokeratin 15 and defines the location of human hair follicle stem cells. *Journal of Cell Science*.

[35] Liu S. H. (2007). *Dissertation*.

[36] Schweizer J., Langbein L., Rogers M. A., Winter H. (2007). Hair follicle-specific keratins and their diseases. *Experimental Cell Research*.

[37] Tong X., Coulombe P. A. (2006). Keratin 17 modulates hair follicle cycling in a TNF-dependent fashion. *Genes & Development*.

[38] McGowan K. M., Tong X., Colucci-Guyon E., Langa F., Babinet C., Coulombe P. A. (2002). Keratin 17 null mice exhibit age- and strain-dependent alopecia. *Genes & Development*.

[39] Kim S., Wong P., Coulombe P. A. (2006). A keratin cytoskeletal protein regulates protein synthesis and epithelial cell growth. *Nature*.

[40] Zhang C., Zhou L., Huang J., Mei X., Wu Z., Shi W. (2018). A preliminary study of growth characteristics of melanocytes co-cultured with keratinocytes in vitro. *Journal of Cellular Biochemistry*.

[41] Fu T., Chai B., Shi Y., Dang Y., Ye X. (2019). Fargesin inhibits melanin synthesis in murine malignant and immortalized melanocytes by regulating PKA/CREB and P38/MAPK signaling pathways. *Journal of Dermatological Science*.

[42] Islam S. M. A., Patel R., Acevedo-Duncan M. (2018). Protein kinase C-*ζ* stimulates colorectal cancer cell carcinogenesis via PKC-*ζ*/Rac1/Pak1/*β*-catenin signaling cascade. *Biochimica et Biophysica Acta (BBA) - Molecular Cell Research*.

[43] Kim D. S., Kim S. Y., Chung J. H., Kim K. H., Eun H. C., Park K. C. (2002). Delayed ERK activation by ceramide reduces melanin synthesis in human melanocytes. *Cellular Signalling*.

[44] Kim E. H., Jeong H. S., Yun H. Y. (2013). Geranylgeranylacetone inhibits melanin synthesis via ERK activation in Mel-Ab cells. *Life Sciences*.

[45] Kim E. H., Kim M. K., Yun H. Y. (2013). Menadione (vitamin K3) decreases melanin synthesis through ERK activation in Mel-Ab cells. *European Journal of Pharmacology*.

[46] Tsegay G., Redi-Abshiro M., Chandravanshi B. S., Ele E., Mohammed A. M., Mamo H. (2020). Effect of altitude of coffee plants on the composition of fatty acids of green coffee beans. *BMC Chemistry*.

[47] Barrera A. (2006). Discussion. *Plastic and Reconstructive Surgery*.

